# PRDM16 Upregulation Induced by MicroRNA-448 Inhibition Alleviates Atherosclerosis via the TGF-β Signaling Pathway Inactivation

This article has been retracted.

**DOI:** 10.3389/fphys.2020.00846

**Published:** 2020-08-11

**Authors:** Dongxing Liu, Jiantao Song, Xianfei Ji, Zunqi Liu, Tao Li, Bo Hu

**Affiliations:** Department of Emergency, Shandong Provincial Hospital Affiliated to Shandong First Medical University, Jinan, China

**Keywords:** microRNA-448, PR domain-containing 16, atherosclerosis, proliferation, apoptosis, migration, oxidative stress, TGF-β signaling pathway

## Abstract

The dysregulated expression of microRNAs (miRs) has been associated with pathological and physiological processes of atherosclerosis (AS). In addition, PR domain-containing 16 (PRDM16), a transcriptional mediator of brown fat cell identity and smooth muscle cell activities, may be involved in the hypercholesterolemia during development of AS. The bioinformatic analysis identified a regulatory miR-448 of PRDM16. Hence, the current study aimed to explore whether miR-448 influenced the activities of aortic smooth muscle cell (ASMCs) in AS. We validated that miR-448 was highly expressed in peripheral blood of patients with AS and aortic smooth muscle of AS model mice. Whereas, PRDM16 was downregulated in the aortic smooth muscle of AS model mice. PRDM16 overexpression was observed to inhibit oxidative stress injury and cell proliferation, and promote apoptosis of ASMCs. Mechanistic studies revealed that miR-448 targeted PRDM16 and negatively regulated the PRDM16 expression, while PRDM16 blocked the TGF-β signaling pathway. Furthermore, Downregulated miR-448 alleviated oxidative stress injury, and attenuated ASMC cell proliferation, migration and enhanced cell apoptosis through upregulation of PRDM16. Taken together, silencing of miR-448 upregulates PRDM16 and inactivates the TGF-β signaling pathway, thereby impeding development of AS by repressing the proliferation, migration and invasion of ASMCs.

## Introduction

Atherosclerosis (AS) is a chronic inflammatory disease characterized by the formation of atherosclerotic plaque in the intima of arteries (Takx et al., 2016). Existing literature has emphasized the distinct effect of smooth muscle cells (SMCs) on the initiation and progression of AS (Doran et al., 2008). The phenotypical transformation of SMCs is a key process in the development of AS (Gomez and Owens, 2012). AS is a primary instigator of coronary artery disease and manifests itself in other conditions including cerebrovascular disease as well as cardiovascular events such as myocardial infarctions, all of which are accompanied by high mortality and morbidity worldwide (Mach et al., 2008; Rader and Daugherty, 2008). Although several therapeutic approaches can be employed for the treatment of AS, there are subgroups of high risk patients who fail to benefit from existing treatment modalities (Ren et al., 2017; Tian et al., 2017).

PR domain containing 16 (PRDM16) is a member of the PR-domain gene family and has been shown to play a role in the pathogenesis of various diseases (Horn et al., 2011). Furthermore, the involvement of PRDM16 has been reported in the regulation of SMC proliferation and differentiation (Davis et al., 2006), suggesting that PRDM16 may participate in the pathogenesis of AS. However, the potential effects of PRDM16 on AS remain largely unknown at present. MicroRNAs (miRs) have been widely documented to regulate various cellular mechanisms, including cytothesis and lipid metabolism, inflammation, as well as the progressive development of AS (Rayner et al., 2012). Mature miRs have been shown to bind to the 3’-untranslated region (3’-UTR) of their target messenger RNAs (mRNAs), inducing the degradation of target mRNAs or inhibiting its translation (Iwakawa and Tomari, 2015). High levels of miR-448 have been underlined in vascular smooth muscle cells (VSMCs) from coronary atherosclerotic plaques, while inhibition of miR-448 has been demonstrated to inhibit the proliferation and migration of VSMCs by targeting MEF2C (Zhang et al., 2017). Moreover, PRDM16 involves in orofacial structures by regulating the transforming growth factor β (TGF-β) signaling pathway (Warner et al., 2007). The inactivation of TGF-β protein expression has also been previously proposed to attenuate reactive oxygen species (ROS)/oxidative stress in AS (Cheng et al., 2019). TGF-β signaling has been reported to suppress AS by inhibiting T cell activation (Robertson et al., 2003). Additionally, the TGF-β signaling pathway plays a regulatory role in SMC activities whereby it helps to inhibit the formation of abdominal aortic aneurysms (Gao et al., 2014), suggesting that the TGF-β signaling may participate in regulating SMCs in AS. Thus, the present work explored potential effects of miR-448 targeting PRDM16 in AS, which may be associated with the TGF-β signaling pathway.

## Materials and Methods

### Ethics Statement

Written informed consent was obtained from all participants prior to the study. Study protocols were approved by the Ethics Committees of Shandong Provincial Hospital Affiliated to Shandong University, based on the ethical principles for medical research involving human subjects of the Helsinki Declaration. Animal experiments were conducted in strict accordance with the Guide to the Management and Use of Laboratory Animals issued by the National Institutes of Health. All procedures related to animal care were conducted under approval of the Institutional Animal Ethics Committee (IAEC No. 39/03/2014).

### miR Prediction

The upstream regulatory miRs of PRDM16 were predicted using the microRNA database^1^, miRSearch database^2^ and TargetScan database^3^. The binding sites between miRs and genes were acquired from the TargetScan database.

### Study Subjects

A total of 158 patients (81 males and 77 females, mean age: 54.66 ± 7.85 years) with moderate-severe AS diagnosed by coronary computed tomographic angiography and coronary angiography in the Department of Cardiology from Shandong Provincial Hospital Affiliated to Shandong University were enrolled. Subjects fasted for 12 h prior to blood collection. Venous blood samples (5 mL) were subsequently obtained on the next morning and then centrifuged at 3000 g for 15 min at room temperature. The upper serum was collected, sub-packed and stored at −80°C for subsequent experiment. Ninety-three serum samples (52 males and 41 females, mean age: 55.71 ± 7.15 years) were collected under controlled conditions from healthy subjects who underwent physical examination serving as normal controls. Clinical data of enrolled patients and healthy subjects are shown in Supplementary Table S1. Reverse transcription quantitative polymerase chain reaction (RT-qPCR) was employed to detect the expression of miR-448 and miR-133b from the respective serum samples.

### Establishment and Identification of AS Mouse Model

A total of 153 male ApoE^–/–^ mice aged 7–8 weeks, weighing 20–25 g were purchased from Beijing Vital River Laboratory Animal Technology Co., Ltd. (Beijing, China). The animals were placed on a controlled standard pelleted diet and provided free access to drinking water. The animals were housed at comfortable controlled room temperature conditions (22 ± 1°C) that were adequately humidified (55 ± 5%). The atherogenic diet was comprised of 10% butterfat, 20% sucrose, 2% cholesterol, and 0.5% cholic acid. Thirty mice were divided into the normal group (*n* = 15) fed with standard food and the AS group (*n* = 15) treated with a 10-week high-fat diet (15% lard, 20% sugar, and 1.2% cholesterol). After 12 weeks, blood samples were collected via retrograde orbital bleeding with the serum subsequently separated. The levels of total cholesterol (TC), triglyceride (TG), and high-density lipoprotein cholesterol (HDL-C) in the serum were measured using a fully automated biochemical analyzer (Beckman Coulter Inc., Fullerton, CA, United States). The mice were euthanized by administering sodium pentobarbital (50 mg/kg), with the aortic tissues of mice dissected and their respective histopathological changes observed and analyzed using hematoxylin-eosin (HE) staining and Oil Red O (ORO) staining methods.

### Production of Lentiviral Particles

A total of 12.5 μg nucleic acid was first diluted into 1 μg/μL with endotoxin-free pure water, and then added with 12.5 μL of water and 25 μL of 10% glucose solution to reach a final volume of 50 μL. Next, 25 μL of Entranster^TM^ (18668-11-1, Engreen, Beijing, China) was diluted with an identical volume of 10% glucose solution culminating with a final volume of 50 μL, followed by the addition of diluted nucleic acid solution which was allowed to rest at room temperature for 15 min. At the fourth week of a high-fat diet, the mice were treated with 50 μL/g (virus titer: 1.0 × 10^13^ viral genome/mL) via intraperitoneal injection of adenovirus-packaged nucleic acid or dimethyl sulfoxide (DMSO) (Ye et al., 2019). After 12 weeks, the mice were euthanized by sodium pentobarbital overdose after which their respective aortas were dissected. The TGF-β signaling pathway inhibitor, LY-364947, was dissolved in 5 mg/mL DMSO solution, diluted with phosphate buffered saline (PBS) and intraperitoneally injected at 1 mg/kg (3 times a week for 3 weeks) (Oka et al., 2008) (Supplementary Figure S1). The mice were classified into the following groups: the overexpressed (oe-) PRDM16 negative control (NC) group (mice infected with lentiviral vector containing oe-PRDM16 NC), the oe-PRDM16 group (mice infected with lentiviral vector containing oe-PRDM16), the miR-448 inhibitor NC group (mice treated with miR-448 inhibitor NC), the miR-448 inhibitor group (mice treated with miR-448 inhibitor), the miR-448 inhibitor + small interfering RNA targeting PRDM16 (si-PRDM16) NC group (mice treated with miR-448 inhibitor and lentiviral vector containing si-PRDM16 NC), the miR-448 inhibitor + si-PRDM16 group (mice treated with miR-448 inhibitor and lentiviral vector containing si-PRDM16), the DMSO group (mice injected with DMSO), and the LY-364947 group (mice injected with TGF-β pathway inhibitor LY-364947).

### Extraction of Aortic Smooth Muscle Cells (ASMCs)

Three mice were selected randomly and placed into the supine position on a small polystyrene foam plate under a dissecting microscope. The chest was cut open to expose the heart and lungs. The aorta was then removed, placed in a 100 mm petri dish, and added with one or two drops of Fungizone solution. Two pairs of forceps were employed to remove the adventitia and obtain a smooth aortic canal. The aorta was then placed into a fresh new 100 mm Petri dish containing one to two drops of the medium. The aorta was cut into square pieces with a side length of approximately 1–2 mm. The aortic mass was placed in a small tissue culture tube containing 100 μL of enzyme solution and incubated in 5% CO_2_ at 37°C for 4–6 h. After gradient suspension and centrifugation, the cells were transferred to a single well of a 48-well plate, placed in 5% CO_2_ at 37°C and permitted to stand for a period of 5 days (Ray et al., 2001).

### HE Staining

The aorta of the mice was fixed, embedded in paraffin, sectioned at a 4-μm thickness, dewaxed with xylene (I) for 5 min, toluene (II) for 5 min, dehydrated using gradient ethanol and subsequently washed with distilled water for 2 min. The sections were then stained using hematoxylin for 5 min, differentiated with hydrochloric acid-ethanol for 30 s, and placed in eosin solution for 2 min. Conventional dehydration, transparency, and blockade with neutral resin were then conducted respectively. Finally, the sections were observed and analyzed under an inverted microscope (XSP-8CA, Shanghai Optical Instrument Factory, Shanghai, China).

### ORO Staining

After the adjacent fat had been removed, the upper part of the thoracic aorta was placed flat on a glass slide, differentiated in 60% isopropanol for 10 min, stained using ORO working solution (ORO:deionized water = 3:2) for 3 h, differentiated in 60% isopropanol for 6–7 times until the background color was observed to have turned white. At last, the image was observed and analyzed using an Olympus digital camera (Olympus Optical Co., Ltd., Tokyo, Japan).

### Immunohistochemistry (IHC)

The paraffin-embedded aortic tissues of the mice were sliced into sections, which were then dewaxed in xylene and hydrated using ethanol of gradient concentrations. Antigen was extracted in citric acid buffer solution. The tissue sections were probed with primary antibodies to intercellular cell adhesion molecule-1 (ICAM-1) (#4915, 1:50, Cell Signaling Technology, Danvers, MA, United States) and vascular cell adhesion molecule-1 (VCAM-1) (ab134047, 1:250, Abcam, Cambridge, United Kingdom) at 4°C overnight. On the next day, sections were re-probed with secondary antibody of goat anti-rabbit antibody to immunoglobulin G (IgG) at 37°C for 20 min and incubated with horseradish peroxidase (HRP)-labeled streptavidin working solution (0343-10000U, Imunbio Co., Ltd., Beijing, China) at 37°C for 20 min. Following development by 3,3’-diaminobenzidine (ST033, Whiga Co., Ltd., Guangzhou, Guangdong, China), sections were counterstained with hematoxylin (PT001, Bogoo Co., Ltd., Shanghai, China) for 1 min. After dehydration by ethanol and clearing by xylene, sections were mounted by neutral resin. Under microscopic observation, five high-power fields were selected from each section on a random basis with 100 cells counted in each field. The percentage of positive cells was calculated.

### Enzyme-Linked Immunosorbent Assay (ELISA)

The levels of malondialdehyde (MDA), superoxide dismutase (SOD), glutathione (GSH) and glutathione peroxidase (GSH-PX) in the cell supernatants were detected using commercially available kits (RAPIDBIO, West Hills, CA, United States). The optical density (OD) value of each well was determined at 450 nm using a Spectramax M5 microplate reader (Molecular Devices, Sunnyvale, CA, United States).

### Detection of ROS Level

The minced aortic tissues of the mice were lysed in order to prepare a single cell suspension, after which the intracellular ROS levels were measured using a peroxide-sensitive fluorescent probe 2’7’-dichlorofluorescein diacetate (DCFH-DA) (Beyotime Biotechnology Inc., Nantong, Jiangsu, China). The cells were exposed to serum-free medium containing 10 μM DCFH-DA for 30 min. Fluorescence was measured using FACSCalibur flow cytometer (Becton-Dickinson, Sunnyvale, CA, United States).

### Dual-Luciferase Reporter Gene Assay

The artificially synthetized PRDM16-3’UTR gene fragments were inserted into pMIR-reporter (Beijing Huayueyang Biotechnology Co., Ltd., Beijing, China) through endonuclease sites SpeI and Hind III. The complementary sequence mutation sites of the seed sequence were designed on the wild-type (WT) PRDM16. The target fragment was subsequently inserted into the pMIR-reporter plasmids by restriction endonuclease digestion using T4 DNA ligase. The correctly sequenced WT and mutant (MUT) plasmids were also co-delivered with miR-448 mimic and mimic NC (GenePhama Co., Ltd., Shanghai, China) into HEK-293T cells (Center for Cell Resources, Shanghai Institute of Life Sciences, Chinese Academy of Sciences, Shanghai, China). Luciferase activity was detected using GloMax 20/20 luminometer (Promega, Madison, WI, United States). The sequences of WT and MUT PRDM16 were as follows: UUAUACAUGAGAUUGAUAUGCAA (WT); TTATACAUTGAGATTGCAGGTACG (MUT).

### 5-Ethynyl-2’-Deoxyuridine (EdU) Assay

The cells (1.6 × 10^5^ cells/well) were incubated with 50 mM EdU (Cell-LightTM EdU Apollo^®^ 488 In Vitro Imaging Kit, Guangzhou Ribobio Biotechnology Co., Ltd., Guangzhou, Guangdong, China) at 37°C for 4 h. The cells were subsequently fixed with 4% formaldehyde for 15 min and treated with 0.5% Triton X-100 for 20 min for permeabilization. The cells were then incubated with 100 mL Apollo^®^ mixture in each well for 30 min, stained with 100 mL Hoechst 33342 dye for 30 min and imaged under a fluorescence microscope (Olympus Corporation, Tokyo, Japan). The number of EdU-positive cells (erythrocytes) was calculated using Image-Pro Plus (IPP) 6.0 software (Media Cybernetics, Bethesda, MD, United States).

### Flow Cytometry

On the next day after transduction, the cells were detached with 0.25% trypsin. The trypsinization process was terminated following the addition of Roswell Park Memorial Institute (RPMI)-1640 medium containing 10% fetal bovine serum. The supernatant was removed through centrifugation at 400 g for 5 min. The cells were fixed with 70% pre-cold ethanol (4°C). The cell density was adjusted to 1 × 10^6^ cells/mL, followed by staining with 10 mL Annexin-V-fluorescein isothiocyanate (FITC)/propidium iodide (PI) (556547, Shanghai Solja Technology Co., Ltd., Shanghai, China) at 4°C for 15–30 min. The cell apoptosis was then detected using a flow cytometer (XL type, conlter, United States). The 525 and 620 nm band-pass filters were excited at 488 nm allowing for FITC and PI fluorescence detection, respectively.

### Immunofluorescence Assay

The cells were fixed with ice-cold acetone and then blocked with 5% (w/v) bovine serum albumin, and incubated with primary antibodies including CD31 (rabbit anti-human, ab28364, 1:20), α-smooth muscle aorta (α-SMA) (rabbit anti-human, ab32575, 1:1000), and vimentin (rabbit anti-human, ab92547, 1:250) overnight at 4°C, followed by incubation with fluorescence-labeled IgG secondary antibody (goat anti-rabbit, 1:200). All antibodies mentioned above were obtained from Abcam. After incubation for 1 h, cells were stained with PI (eBioscience, San Diego, CA, United States), mounted, and visualized using fluorescence microscopy (Olympus IX51, Tokyo, Japan).

### Scratch Assay

Horizontal lines were drawn on the back of the 6-well plate. The cells were trypsinized with 0.25% trypsin and triturated into a single cell suspension. The cells were then counted and inoculated into a 6-well plate at 1 × 10^6^ cells/well. Following a 24-h period of incubation, the cells were cultured in RPMI 1640 medium. An artificial scratch was then made with the sterile 10 μL micropipette tip. The cells detached on the tip of the pipette were then removed. The remaining cells were then cultured in serum-free medium at 37°C with 5% CO_2_. Photographs were taken at 0 h and at 48 h under a microscope (Olympus Corporation, Tokyo, Japan).

### RT-qPCR

Total RNA was extracted and reversely transcribed into cDNA. The primers were designed and submitted to Sangon Biotech (Shanghai, China) for design and synthesis (Table 1). The RT-qPCR assay was performed by EasyScript First-Strand cDNA Synthesis SuperMix (Catalog No. AE301-02, TransGen Biotech, Beijing, China). Fluorescent qPCR was conducted using SYBR^®^ Premix Ex Taq^TM^ II Kit (TaKaRa, Dalian, Liaoning, China). RT-qPCR assays were performed using the ABI’s 7500-type real-time PCR. Gene expression was detected using 2^–ΔΔCt^.

**TABLE 1:** Primer sequences for RT-qPCR.

**Targeted genes**	**Primer sequences**
miR-448	F: 5′-TTATTGCGATGTGTTCCTTATG-3′
	R: 5′-ATGCATGCCACGGGCATATACACT-3′
miR-133b	F: 5′-GCGCTTTGGTCCCCTTC-3′
	R: 5′-CAGTGCAGGGTCCGAGGT-3′
PRDM16	F: 5′-CCACCAGCGAGGACTTCAC-3′
	R: 5′-GGAGGACTCTCGTAGCTCGAA-3′
TGF-β	F: 5′-CCACCTGCAAGACCATCGAC-3′
	R: 5′-CTGGCGAGCCTTAGTTTGGAC-3′
Smad2	F: 5′-AAGCCATCACCACTCAGAATTG-3′
	R: 5′-CACTGATCTACCGTATTTGCTGT-3′
Smad3	F: 5′-AGGGGCTCCCTCACGTTATC-3′
	R: 5′-CATGGCCCGTAATTCATGGTG-3′
U6	F: 5′-CTCGCTTCGGCAGCACA-3′
	R: 5′-AACGCTTCACGAATTTGCGT-3′
GAPDH	F: 5′-GGAGCGAGATCCCTCCAAAAT-3′
	R: 5′-GGCTGTTGTCATACTTCTCATGG-3′

*F, forward; R, reverse; miR-448, microRNA-448; miR-133b, microRNA-133b; PRDM16, PR domain containing 16; TGF-β, transforming growth factor β; Smad2, SMAD family member 2; Smad3, SMAD family member 3; RT-qPCR, reverse transcription quantitative polymerase chain reaction; GAPDH, glyceraldehyde-3-phosphate dehydrogenase.*

### Western Blot Analysis

The total tissues and cells were lysed using radio-immunoprecipitation assay (RIPA) lysis buffer (P0013B, Beyotime Biotechnology Co., Ltd., Shanghai, China), and added with phenylmethylsulfonyl fluoride (PMSF) and phosphatase inhibitor to collect total protein, which was separated by sodium dodecyl sulfate-polyacrylamide gel electrophoresis and transferred onto the nitrocellulose membrane. The membrane was then incubated with the primary antibodies at 4°C overnight: PRDM16 (rabbit, ab106410, 1:1000), TGF-β (rabbit, ab92486, 1:2000), Smad2 (rabbit, ab33875, 1:1000), phosphorylated (p)-SMAD family member 2 (Smad2) (rabbit, ab53100, 1:1000), SMAD family member 3 (Smad3) (rabbit, ab40854, 1:1000), p-Smad3 (rabbit, a52903, 1:2000), and glyceraldehyde-3-phosphate dehydrogenase (GAPDH) (rabbit anti-human, ab9485, 1:2500). All antibodies and dilutions were purchased from Abcam. After blocking, the membrane was probed using diluted HRP-labeled secondary antibody IgG (goat anti-rabbit, ab205718, 1:5000), and then incubated for 2 h. The membrane was visualized by enhanced chemiluminescence using the SmartView Pro 2000 (UVCI-2100, Major Science, United States). The gray value ratio of protein was analyzed using Quantity One software.

### Statistical Analysis

Statistical analyses were performed using SPSS 21.0 statistical software (IBM Corp. Armonk, NY, United States). All measurement data were expressed as mean ± standard deviation. The data of two groups with normal distribution and equal variance were compared by unpaired *t*-test. A *p* < 0.05 value was regarded as being of statistical significance.

## Results

### miR-448 Was Highly Expressed While PRDM16 Was Poorly Expressed in AS Patients and Mice

In order to elucidate the regulatory mechanism by which the PRDM16 gene influences AS, the upstream regulatory miRs of PRDM16 were predicted by such databases as microRNA, miRSearch and TargetScan, and the intersection of the predicted results was obtained. Among the database predicted results, two miRs (miR-448 and miR-133b) were considered to target PRDM16 (Figure 1A). Quantitative analyses revealed that miR-448 was highly expressed in the serum of patients with AS (Figure 1B). Further prediction of the targeted binding sites between miR-448 and PRDM16 in mice and humans illustrated that miR-448 might target PRDM16, while the sequence of miR-448 and its binding site to the gene were almost identical in both human and mice forms (Figure 1C), suggesting that miR-448 may participate in AS in mice by targeting PRDM16.

**FIGURE 1:** miR-448 was upregulated while PRDM16 was downregulated in AS patients and mice. **(A)** The intersection of PRDM16 upstream miRs predicted by MicroRNA and other databases. The three circles in the figure represent the prediction results of three databases for PRDM16, while the overlapped part represents the intersection of three databases. **(B)** RT-qPCR results of miR-448 and miR-133b in serum from 158 AS samples and 93 normal samples. **(C)** Targeted binding site prediction of PRDM16 and miR-448 in human and mice. **(D)** The quantitative analysis of TC, TG, and HDL-C in peripheral blood of mice. **(E)** The content of oxidative stress-related indicators (MDA, SOD, GSH, and GSH-PX) as detected by ELISA. **(F)** ROS levels in mice serum. **(G)** The number of aortic thrombosis in AS mice as detected by ORO staining (×400, scale bar: 25 μm). **(H)** The aortic plaque changes in AS mice as detected by HE staining (×200, scale bar: 50 μm). **(I)** The relative expression of miR-448 and PRDM16 in mice aorta as detected by RT-qPCR. **(J)** PRDM16 protein expression in mice aorta as detected by Western blot analysis. **(K)** Gray value quantitation of panel **(J)**. * *p* < 0.05 compared with normal samples. The measurement data were expressed as mean ± standard deviation, and the data were analyzed by independent-sample *t*-test, *n* = 15.

Following the successful AS mouse model establishment, biochemical indicators (Figure 1D) and ELISA for oxidative stress-related indicators (Figures 1E,F) demonstrated that in comparison with the normal mice, the levels of TC, TG, MDA and ROS were upregulated, while the HDL-C, SOD, GSH, and GSH-PX levels were downregulated in mice with AS (*p* < 0.05). Both ORO staining (red staining area: the thrombus block) and HE staining (the achromatic block-like area: AS plaque) revealed that the numbers of thrombi and AS plaque were dramatically elevated in the aortic tissues of mice with AS when compared with the normal tissues (*p* < 0.05) (Figures 1G,H). RT-qPCR and Western blot analysis results demonstrated that the expression of miR-448 was upregulated while that of PRDM16 was downregulated in the aortic smooth muscle of mice with AS when compared with the normal mice (*p* < 0.05) (Figures 1I–K). Based on the aforementioned analysis results, it was concluded that miR-448 was highly expressed while PRDM16 was poorly expressed in AS, indicating that miR-448 and PRDM16 may participate in the regulation of AS.

### Overexpressed PRDM16 Inhibited Oxidative Stress Injury and ASMC Proliferation While Promoting Cell Apoptosis

Next, we set out to further investigate the biological function of PRDM16 on ASMCs in AS mice and normal mice. The ELISA detection results regarding the oxidative stress-related indicators (Supplementary Figures S2A,B), EdU proliferation assay (Figures 2A,B), and flow cytometry apoptosis assay (Figures 2C,D) demonstrated that there had been a distinct downregulation of MDA and ROS levels, remarkable upregulation of SOD, GSH, and GSH-PX levels, notably diminished cell proliferation, as well as an obvious elevation in cell apoptosis in the supernatant of ASMCs of the oe-PRDM16 group compared with its NC (*p* < 0.05). The immunofluorescence detection results (Figures 2E,F) and scratch assay results (Figures 2G,H) indicated that in comparison with corresponding NC, fluorescence intensity of CD31 in response to oe-PRDM16 was increased, while α-SMA, vimentin and cell migration were all reduced (all *p* < 0.05). As shown in Figures 2I–K, compared with oe-PRDM16 NC, the expression of PRDM16 was increased in cells transduced with oe-PRDM16 (*p <* 0.05). In conclusion, PRDM16 overexpression can inhibit oxidative stress injury and cell proliferation, and promote apoptosis of ASMCs.

**FIGURE 2:** Overexpression of PRDM16 suppressed proliferation of ASMCs while enhancing apoptosis in AS mice. **(A)** EdU proliferation staining of cells in each group (×200, scale bar: 50 μm). **(B)** The relative fold of EdU positive cell in each group. **(C)** The apoptosis of cells in each group as detected by flow cytometry. **(D)** The apoptosis rate in each group as detected by flow cytometry. **(E)** Immunofluorescence of cells in each group (×200, scale bar: 50 μm), green staining was regarded as positive results. **(F)** The fluorescence intensity of CD31, α-SMA, and vimentin of cells in each group. **(G)** The cell migration in each group as detected by scratch assay. **(H)** The relative migration in each group. **(I)** The relative expression of miR-448 and PRDM16 as detected by RT-qPCR. **(J,K)** The expression of PRDM16 protein normalized to GAPDH as detected by Western blot analysis. *p < 0.05 compared with ASMCs transduced with oe-PRDM16 NC. The measurement data were expressed as mean ± standard deviation, and analyzed by independent-sample *t*-test, and the experiment was repeated three times independently.

### Silencing of miR-448 Upregulates PRDM16 to Inhibit Oxidative Stress Injury, Cell Proliferation, Migration, and Invasion While Promoting Apoptosis of ASMCs

As illustrated in Figure 3A, dual luciferase reporter gene assay revealed that luciferase activity of PRDM16-WT was decreased in cells transduced with miR-448 mimic when compared with its NC (*p* < 0.05), with no significant change detected in PRDM16-MUT (*p* > 0.05), indicating that miR-448 could target PRDM16.

**FIGURE 3:** Silencing of miR-448 inhibited the cell proliferation, migration, and invasion while promoting the apoptosis of ASMCs by upregulating the expression of PRDM16. **(A)** The relative luciferase activity of miR-448 and PRDM16, *p < 0.05 compared with the NC group. **(B)** ROS levels of cells in each group. **(C)** Representative images of EdU proliferation staining of cells in each group (×200, scale bar: 50 μm). **(D)** The relative fold of EdU positive cell in each group. **(E)** The apoptosis of cells in each group as detected by flow cytometry. **(F)** The apoptosis rate in each group as detected by flow cytometry. **(G)** Immunofluorescence of cells in each group (×200, scale bar: 50 μm). **(H)** The fluorescence intensity of CD31, α-SMA, and vimentin of cells in each group. **(I)** The cell migration in each group as detected by scratch assay. **(J)** The relative migration in each group. **(K)** The relative expression of miR-448 and PRDM16 as detected by RT-qPCR. **(L,M)** The expression of PRDM16 protein normalized to GAPDH as detected by Western blot analysis. *p < 0.05 compared with ASMCs transduced with miR-448 inhibitor NC, ^#^*p* < 0.05 compared with ASMCs transduced with miR-448 inhibitor + si-PRDM16 NC. The measurement data were expressed as mean ± standard deviation, and the data of two groups were analyzed by independent-sample *t*-test. The experiment was repeated three times independently.

Next, to further verify the effects of miR-448 and PRDM16 on the biological functions of ASMCs, ELISA (Figure 3B and Supplementary Figure S3), EdU proliferation assay (Figures 3C,D), flow cytometry assay (Figures 3E,F), immunofluorescence assay (Figures 3G,H), and scratch assay (Figures 3I,J) were performed, respectively. The results demonstrated that compared with cells transduced with miR-448 inhibitor NC, the MDA and ROS levels were downregulated while SOD, GSH, and GSH-PX levels were upregulated in cells transduced with miR-448 inhibitor, also, cell proliferation and migration were diminished while apoptosis was increased, the levels of CD31 expression were increased, while α-SMA and vimentin were decreased (*p* < 0.05). There was no significant difference detected regarding the levels of MDA, SOD, GSH, GSH-PX, ROS, cell proliferation, migration and apoptosis, CD31, α-SMA, and vimentin in cells transduced with miR-448 inhibitor + si-PRDM16 (*p* > 0.05). Relative to cells transduced with miR-448 inhibitor + si-PRDM16 NC, MDA, and ROS levels in cells transduced with miR-448 inhibitor + si-PRDM16 were upregulated while SOD, GSH, and GSH-PX levels were downregulated; cell proliferation and migration were increased while cell apoptosis was decreased; CD31 expression was decreased while α-SMA and vimentin expression was increased (*p* < 0.05).

As shown in Figures 3K–M, the expression of miR-448 was decreased while PRDM16 expression was increased in cells transduced with miR-448 inhibitor when compared with cells transduced with miR-448 inhibitor NC (all *p* < 0.05). The expression of miR-448 in cells transduced with miR-448 inhibitor + si-PRDM16 was decreased (*p* < 0.05). Relative to cells transduced with miR-448 inhibitor + si-PRDM16 NC, PRDM16 expression was decreased (*p* < 0.05), while the expression of miR-448 remained unchanged in cells transduced with miR-448 inhibitor + si-PRDM16. Therefore, miR-448 inhibition can upregulate the expression of PRDM16, thus inhibiting oxidative stress injury, cell proliferation, migration and invasion, but promoting apoptosis of ASMCs.

### PRDM16 Inactivated the TGF-β Signaling Pathway to Inhibit Oxidative Stress Injury, Proliferation, Migration, and Invasion of ASMCs While Promoting Apoptosis

The regulatory role of PRDM16 in TGF-β2 signaling pathway was previously explored from a hematopoiesis perspective (Avagyan et al., 2011). The inactivation of the protein expression of TGF-β was also proposed as an approach to restrict ROS in AS (Jones et al., 2009). Thus, we speculated that PRDM16 could be involved in the development of AS and act to regulate the TGF-β signaling pathway. The ELISA regarding oxidative stress-related indicators (Supplementary Figures S4A,B), EdU proliferation assay (Figures 4A,B), flow cytometry assay (Figures 4C,D), immunofluorescence assay (Figures 4E,F), and scratch assay (Figures 4G,H) demonstrated that, when compared with mice treated with DMSO, mice treated with LY-364947 exhibited downregulated MDA and ROS levels, upregulated levels of SOD, GSH, and GSH-PX, restricted ASMC proliferation and migration and accelerated apoptosis, along with elevated CD31 level and diminished levels of α-SMA and vimentin (*p* < 0.05). Relative to mice treated with oe-PRDM16 NC, MDA, and ROS levels were downregulated, while SOD, GSH, and GSH-PX levels were upregulated, cell proliferation, and migration were diminished while apoptosis was increased, CD31 expression was enhanced, while α-SMA and vimentin were suppressed in mice treated with oe-PRDM16 (*p* < 0.05).

**FIGURE 4:** Overexpressed PRDM16 inhibited the cell proliferation, migration, and invasion while promoting the apoptosis of ASMCs by inactivation of the TGF-β signaling pathway. **(A)** Representative images of EdU proliferation staining of cells in each group (×200, scale bar: 50 μm). **(B)** The relative fold of EdU positive cell in each group. **(C)** The apoptosis of cells in each group as detected by flow cytometry. **(D)** The apoptosis rate in each group as detected by flow cytometry. **(E)** Immunofluorescence of cells in each group (×200, scale bar: 50 μm). **(F)** The fluorescence intensity of CD31, α-SMA, and vimentin of cells in each group. **(G)** The cell migration in each group as detected by scratch assay. **(H)** The relative migration in each group. **(I)** The relative expression of PRDM16, TGF-β, p-Smad2, and p-Smad3 as detected by RT-qPCR. **(J,K)** The expression of PRDM16 protein normalized to GAPDH as detected by Western blot analysis. *p < 0.05 compared with ASMCs treated with DMSO, ^#^*p* < 0.05 compared with ASMCs treated with oe-PRDM16 NC. The measurement data were expressed as mean ± standard deviation, and analyzed by independent-sample *t*-test. The experiment was repeated three times independently.

As illustrated in Figures 4I–K, when compared with mice treated with DMSO, the extent of Smad2 and Smad3 phosphorylation in the LY-364947-treated mice was decreased (*p* < 0.05). Relative to mice treated with oe-PRDM16 NC, the expression of PRDM16 in mice treated with oe-PRDM16 was elevated while the expression of TGF-β, and extent of Smad2 and Smad3 phosphorylation were decreased (*p* < 0.05). In a word, PRDM16 overexpression can block the TGF-β signaling pathway, thereby inhibiting oxidative stress injury, cell proliferation, migration and invasion while promoting apoptosis of ASMCs.

### PRDM16 Impeded AS by Inhibiting the Activation of the TGF-β Signaling Pathway *in vivo*

In order to clarify the effects of PRDM16 and the downstream TGF-β signaling pathway on the progression of AS, the AS mice were transduced with LY-364947 or oe-PRDM16. The results of biochemical indicators (Figure 5A), HE staining (Figure 5B), ORO staining (Figure 5C), and IHC (Figure 5D) illustrated that, vs. mice treated with DMSO, TC and TG levels were downregulated and positive rate of AS markers (ICAM-1 and VCAM-1) reduced in mice treated with LY-364947, which also displayed upregulated HDL-C levels, and reduced number of AS plaques and thrombi in the aortic tissues (all *p* < 0.05). Relative to mice treated with oe-PRDM16 NC, TC, and TG levels were downregulated and positive rate of AS markers (ICAM-1 and VCAM-1) reduced in mice treated with oe-PRDM16, which also exhibited upregulated HDL-C levels, and diminished number of AS plaques and thrombi in the aortic tissues (*p* < 0.05). The aforementioned results demonstrated that PRDM16 suppresses activation of the TGF-β signaling pathway to halt the progression of AS in mice.

**FIGURE 5:** PRDM16 inhibited AS through inactivation of the TGF-β signaling pathway. **(A)** The content of TC, TG, and HDL-C in peripheral blood in mice in each group as detected by biochemical indicators. **(B)** The changes of aortic plaques in AS mice as detected by HE staining (×200, scale bar: 50 μm). **(C)** The number of aortic thrombosis in AS mice as detected by ORO staining (×400, scale bar: 25 μm). **(D)** Positive rates of AS markers (ICAM-1 and VCAM-1) in the aorta of AS mice as detected by IHC (×400). *p < 0.05 compared with mice treated with DMSO, ^#^*p* < 0.05 compared with mice treated with oe-PRDM16 NC. The measurement data were expressed as mean ± standard deviation, and analyzed by independent-sample *t*-test, *n* = 15.

## Discussion

AS is a complicated multi-factor disease associated with various risk factors, including arterial hypertension, dyslipidemia, diabetes mellitus, and smoke (Fava and Montagnana, 2018). Thus, the identification of novel therapeutic targets is of urgent need in order to facilitate the diagnosis and treatment of patients with AS. In the present study, we investigated that inhibition of miR-448 could potentially prevent AS development *via* inactivation of the TGF-β signaling pathway by targeting PRDM16.

PRDM16 exhibited downregulated levels in the serum samples of both AS patients as well as the aortic smooth muscle of AS mouse models. Overexpressed PRDM16 was found to restrict ASMC oxidative stress injury, proliferation and migration, while acting to enhance apoptosis. The dysregulation of PRDM16 has been implicated in the progression of various diseases (Kinameri et al., 2008; Zhu et al., 2017). The ectopic expression of PRDM16 has been shown to promote the trans-differentiation of VSMCs into beige adipocytes, indicating that PRDM16 may regulate development of AS through VSMCs (Brown et al., 2014). Evidence exists reporting that overexpression of PRDM16 decreases the levels of ROS (Chuikov et al., 2010). Decreased levels of SOD, GSH and GSH-Px and increased MDA levels were indicative of aggravated oxidative stress damage (Zhao et al., 2018). Therefore, PRDM16 overexpression could curb oxidative stress. Interestingly, PRDM16 is a transcriptional mediator of brown fat cell identity (Kajimura et al., 2010) and brown fat like gene expression is correlated with HDL-C and TC levels in coronary artery disease (Gautron, 2015). Further, brown fat activation attenuates hypercholesterolaemia and prevents development of AS (Berbee et al., 2015). Moreover, decreased contents of TC, and TG, along with increased contents of HDL-C can be indicative of the attenuated AS (Wang et al., 2018). Thus, PRDM16 overexpression could impede lipid accumulation in AS, and PRDM16 downregulation-induced by miR-448 accelerated development of AS. CD31, also known as platelet/endothelial cell adhesion molecule-1, has been elucidated to be expressed at a high level at endothelial cell-cell junctions to maintain the integrity and accelerate the recovery of the vascular permeability barrier in response to inflammatory or thrombotic challenge (Liu and Shi, 2012; Lertkiatmongkol et al., 2016). Additionally, a functional study has deciphered that α-SMA-positive VSMCs appreciably elevated in the progression of AS (Zhu et al., 2019). Also, Vimentin has been recognized as an indicator of cell migration, and loss of vimentin triggers enhanced oxidative stress and promoted vascular inflammation in macrophages, alleviating AS in a mouse model (Battaglia et al., 2018; Haversen et al., 2018). Accordingly, ectopic PRDM16 expression could attenuate oxidative stress injury and lipid accumulation, as evidenced by the elevated levels of CD31, HDL-C, SOD, GSH and GSH-Px and decreased levels of α-SMA, vimentin, TC, TG, MDA. Besides, miR-448-mediated PRDM16 inhibition accelerated development of AS.

Notably, PRDM16 was targeted and negatively regulated by miR-448. miR-448 was upregulated in serum samples of AS patients and AS mice, and its silencing inhibited ASMC oxidative stress injury, proliferation, and migration. Previous studies have demonstrated that miR-448 is upregulated in VSMCs of coronary atherosclerotic plaques, while the inhibition of miR-448 suppresses oxidative stress injury, proliferation, and migration of VSMCs by targeting MEF2C (Zhang et al., 2017). There is an accumulating amount of evidence suggesting that multiple miRs may regulate PRDM16 in various diseases. For instance, inhibition of miR-133 has been shown to trigger upregulation of thermogenesis and energy expenditure by targeting PRDM16 (Liu and Kuang, 2013). Besides, miR-133 has been reported to inhibit the brown adipose determination by targeting PRDM16 (Yin et al., 2013). Moreover, PRDM16 inhibited AS by blocking the TGF-β signaling pathway. The TGF-β signaling pathway shares a strong association with migration and proliferation of SMCs, as well as AS progression (Zhao et al., 2019). Prior evidence also revealed that PRDM16 could exert its regulation through the TGF signaling pathway (Avagyan et al., 2011). Besides, the activation of the TGF-β signaling pathway has been reported to elevate oxidative stress as well as the levels of ROS in AS (Cheng et al., 2019). Thus, downregulation of PRDM16 induced by miR-448 activated the TGF-β signaling pathway, which ultimately influenced the development of AS. Of note, multiple miRs have been suggested to harbor clinical application value for AS (Qin et al., 2018; Han et al., 2019; Li et al., 2019; Liu et al., 2019), highly suggestive of the therapeutic implication of miR-448 as a physiologically validated approach for the prevention and treatment of AS.

## Conclusion

Taken together, inhibition of miR-448 upregulated the expression of PRDM16 thereby inactivating the TGF-β signaling pathway, which suppressed the oxidative stress injury, proliferation and migration of ASMCs. The present study provides evidence highlighting the involvement of the miR-448/PRDM16/TGF-β axis in the pathophysiological process of AS. However, further investigations are required into the modulation of miR-448 and its downstream targets, which may be a novel therapeutic and diagnostic strategy for AS.

## Data Availability Statement

The raw data supporting the conclusions of this article will be made available by the authors, without undue reservation, to any qualified researcher.

## Ethics Statement

Written informed consent was obtained from all participants prior to the study. Study protocols were approved by the Ethics Committees of the Shandong Provincial Hospital Affiliated to Shandong University and based on the ethical principles for medical research involving human subjects of the Helsinki Declaration. Animal experiments were conducted in strict accordance with the Guide to the Management and Use of Laboratory Animals issued by the National Institutes of Health. All procedures related to animal care were conducted under approval of the Institutional Animal Ethics Committee (IAEC No. 39/03/2014).

## Author Contributions

DL designed the study. DL and JS collated the data. DL, XJ, and ZL analyzed and produced the initial draft of the manuscript. TL and BH contributed to the drafting of the manuscript. All authors contributed to the article and approved the submitted version.

## Conflict of Interest

The authors declare that the research was conducted in the absence of any commercial or financial relationships that could be construed as a potential conflict of interest.

## Footnotes

1
http://www.microrna.org/microrna/home.do?tdsourcetag=s_pcqq_aiomsg

2
https://www.exiqon.com/miRSearch

3
http://www.targetscan.org/vert_71/

## Supplementary Material

FIGURE S1 The flow diagram depicting the development of AS model in mice. **(A)** Normal mice on standard diet. **(B)** ApoE^–/–^ mice on atherogenic diet for 10 weeks to induce AS. **(C)** Adenovirus or TGF-β inhibitor (LY-364947) was intraperitoneally injected into ApoE^–/–^ mice on atherogenic diet from the 4th week, 3 times a week for 3 weeks.

FIGURE S2 Overexpression of PRDM16 suppressed oxidative stress injury of ASMCs in AS mice. **(A)** The content of oxidative stress-related indicators (MDA, SOD, GSH, and GSH-PX) in each group of cell supernatant as detected by ELISA. **(B)** ROS levels in cells in each group. ^∗^*p* < 0.05 compared with ASMCs transduced with oe-PRDM16 NC. The measurement data were expressed as mean ± standard deviation, and analyzed by independent-sample *t*-test, and the experiment was repeated three times independently.

FIGURE S3 Silencing of miR-448 inhibited the oxidative stress injury of ASMCs by up-regulating the expression of PRDM16. The content of oxidative stress-related indicators (MDA, SOD, GSH, and GSH-PX) in the cell supernatant was measured by ELISA. ^∗^*p* < 0.05 compared with ASMCs transduced with miR-448 inhibitor NC, ^#^*p* < 0.05 compared with ASMCs transduced with miR-448 inhibitor + si-PRDM16 NC. The measurement data were expressed as mean ± standard deviation, and analyzed by independent-sample *t*-test between two groups. The experiment was repeated three times independently.

FIGURE S4 Overexpressed PRDM16 inhibited the oxidative stress injury of ASMCs by inactivation of the TGF-β signaling pathway. **(A)** The content of oxidative stress-related indicators (MDA, SOD, GSH, and GSH-PX) as detected by ELISA. **(B)** ROS levels of cells in each group. ^∗^*p* < 0.05 compared with ASMCs treated with DMSO, ^#^*p* < 0.05 compared with ASMCs treated with oe-PRDM16 NC. The measurement data were expressed as mean ± standard deviation, and analyzed by independent-sample *t*-test. The experiment was repeated three times independently.

## References

[B1] AvagyanS.AguiloF.KamezakiK.SnoeckH. W. (2011). Quantitative trait mapping reveals a regulatory axis involving peroxisome proliferator-activated receptors, PRDM16, transforming growth factor-beta2 and FLT3 in hematopoiesis. *Blood* 118 6078–6086. 10.1182/blood-2011-07-365080 21967974PMC3234666

[B2] BattagliaR. A.DelicS.HerrmannH.SniderN. T. (2018). Vimentin on the move: new developments in cell migration. *F1000Res.* 7:1796. 10.12688/f1000research.15967.1 30505430PMC6241562

[B3] BerbeeJ. F.BoonM. R.KhedoeP. P.BarteltA.SchleinC.WorthmannA. (2015). Brown fat activation reduces hypercholesterolaemia and protects from atherosclerosis development. *Nat. Commun.* 6:6356. 10.1038/ncomms7356 25754609PMC4366535

[B4] BrownN. K.ZhouZ.ZhangJ.ZengR.WuJ.EitzmanD. T. (2014). Perivascular adipose tissue in vascular function and disease: a review of current research and animal models. *Arterioscl. Thromb. Vasc. Biol.* 34 1621–1630. 10.1161/ATVBAHA.114.303029 24833795PMC4104287

[B5] ChengY.ZhouM.ZhouW. (2019). MicroRNA-30e regulates TGF-beta-mediated NADPH oxidase 4-dependent oxidative stress by Snai1 in atherosclerosis. *Int. J. Mol. Med.* 43 1806–1816. 10.3892/ijmm.2019.4102 30816428PMC6414159

[B6] ChuikovS.LeviB. P.SmithM. L.MorrisonS. J. (2010). Prdm16 promotes stem cell maintenance in multiple tissues, partly by regulating oxidative stress. *Nat. Cell Biol.* 12 999–1006. 10.1038/ncb2101 20835244PMC2948585

[B7] DavisC. A.HaberlandM.ArnoldM. A.SutherlandL. B.McDonaldO. G.RichardsonJ. A. (2006). PRISM/PRDM6, a transcriptional repressor that promotes the proliferative gene program in smooth muscle cells. *Mol. Cell Biol.* 26 2626–2636. 10.1128/MCB.26.7.2626-2636.2006 16537907PMC1430312

[B8] DoranA. C.MellerN.McNamaraC. A. (2008). Role of smooth muscle cells in the initiation and early progression of atherosclerosis. *Arterioscler. Thromb. Vasc. Biol.* 28 812–819. 10.1161/ATVBAHA.107.159327 18276911PMC2734458

[B9] FavaC.MontagnanaM. (2018). Atherosclerosis is an inflammatory disease which lacks a common anti-inflammatory therapy: how human genetics can help to this issue. a narrative review. *Front. Pharmacol.* 9:55. 10.3389/fphar.2018.00055 29467655PMC5808208

[B10] GaoF.ChambonP.OffermannsS.TellidesG.KongW.ZhangX. (2014). Disruption of TGF-beta signaling in smooth muscle cell prevents elastase-induced abdominal aortic aneurysm. *Biochem. Biophys. Res. Commun.* 454 137–143. 10.1016/j.bbrc.2014.10.053 25450370

[B11] GautronL. (2015). Toward a neuroimmunoendocrinology of adipose tissue. *Endocrinology* 156 3485–3487. 10.1210/en.2015-1735 26380935PMC4588829

[B12] GomezD.OwensG. K. (2012). Smooth muscle cell phenotypic switching in atherosclerosis. *Cardiovasc. Res.* 95 156–164. 10.1093/cvr/cvs115 22406749PMC3388816

[B13] HanZ.GuanY.LiuB.LinY.YanY.WangH. (2019). MicroRNA-99a-5p alleviates atherosclerosis via regulating Homeobox A1. *Life Sci.* 232:116664. 10.1016/j.lfs.2019.116664 31325426

[B14] HaversenL.SundelinJ. P.MardinogluA.RutbergM.StahlmanM.WilhelmssonU. (2018). Vimentin deficiency in macrophages induces increased oxidative stress and vascular inflammation but attenuates atherosclerosis in mice. *Sci. Rep.* 8:16973. 10.1038/s41598-018-34659-2 30451917PMC6242955

[B15] HornK. H.WarnerD. R.PisanoM.GreeneR. M. (2011). PRDM16 expression in the developing mouse embryo. *Acta Histochem.* 113 150–155. 10.1016/j.acthis.2009.09.006 19853285PMC2891916

[B16] IwakawaH. O.TomariY. (2015). The functions of microRNAs: mRNA decay and translational repression. *Trends Cell Biol.* 25 651–665. 10.1016/j.tcb.2015.07.011 26437588

[B17] JonesJ. A.SpinaleF. G.IkonomidisJ. S. (2009). Transforming growth factor-beta signaling in thoracic aortic aneurysm development: a paradox in pathogenesis. *J. Vasc. Res*. 46, 119–137. 10.1159/000151766 18765947PMC2645475

[B18] KajimuraS.SealeP.SpiegelmanB. M. (2010). Transcriptional control of brown fat development. *Cell Metab.* 11 257–262. 10.1016/j.cmet.2010.03.005 20374957PMC2857670

[B19] KinameriE.InoueT.ArugaJ.ImayoshiI.KageyamaR.ShimogoriT. (2008). Prdm proto-oncogene transcription factor family expression and interaction with the Notch-Hes pathway in mouse neurogenesis. *PLoS One* 3:e3859. 10.1371/journal.pone.0003859 19050759PMC2585159

[B20] LertkiatmongkolP.LiaoD.MeiH.HuY.NewmanP. J. (2016). Endothelial functions of platelet/endothelial cell adhesion molecule-1 (CD31). *Curr. Opin. Hematol.* 23 253–259. 10.1097/MOH.0000000000000239 27055047PMC4986701

[B21] LiY.YangN.DongB.YangJ.KouL.QinQ. (2019). MicroRNA-122 promotes endothelial cell apoptosis by targeting XIAP: therapeutic implication for atherosclerosis. *Life Sci.* 232:116590. 10.1016/j.lfs.2019.116590 31228514

[B22] LiuL.ShiG. P. (2012). CD31: beyond a marker for endothelial cells. *Cardiovasc. Res.* 94 3–5. 10.1093/cvr/cvs108 22379038

[B23] LiuQ. Q.RenK.LiuS. H.LiW. M.HuangC. J.YangX. H. (2019). MicroRNA-140-5p aggravates hypertension and oxidative stress of atherosclerosis via targeting Nrf2 and Sirt2. *Int. J. Mol. Med.* 43 839–849. 10.3892/ijmm.2018.3996 30483753PMC6317688

[B24] LiuW.KuangS. (2013). miR-133 links to energy balance through targeting Prdm16. *J. Mol. Cell. Biol.* 5 432–434. 10.1093/jmcb/mjt036 24085747PMC3900862

[B25] MachF.MontecuccoF.SteffensS. (2008). Cannabinoid receptors in acute and chronic complications of atherosclerosis. *Br. J. Pharmacol.* 153 290–298. 10.1038/sj.bjp.0707517 17965744PMC2219535

[B26] OkaM.IwataC.SuzukiH. I.KiyonoK.MorishitaY.WatabeT. (2008). Inhibition of endogenous TGF-beta signaling enhances lymphangiogenesis. *Blood* 111 4571–4579. 10.1182/blood-2007-10-120337 18310502

[B27] QinB.ShuY.LongL.LiH.MenX.FengL. (2018). MicroRNA-142-3p induces atherosclerosis-associated endothelial cell apoptosis by directly targeting rictor. *Cell. Physiol. Biochem.* 47 1589–1603. 10.1159/000490932 29949787

[B28] RaderD. J.DaughertyA. (2008). Translating molecular discoveries into new therapies for atherosclerosis. *Nature* 451 904–913. 10.1038/nature06796 18288179

[B29] RayJ. L.LeachR.HerbertJ. M.BensonM. (2001). Isolation of vascular smooth muscle cells from a single murine aorta. *Methods Cell Sci.* 23 185–188. 10.1023/a:101635751014312486328

[B30] RaynerK. J.Fernandez-HernandoC.MooreK. J. (2012). MicroRNAs regulating lipid metabolism in atherogenesis. *Thromb. Haemost.* 107 642–647. 10.1160/TH11-10-0694 22274626PMC3618663

[B31] RenY.QiaoW.FuD.HanZ.LiuW.YeW. (2017). Traditional chinese medicine protects against cytokine production as the potential immunosuppressive agents in atherosclerosis. *J. Immunol. Res.* 2017:7424307. 10.1155/2017/7424307 29038791PMC5606136

[B32] RobertsonA. K.RudlingM.ZhouX.GorelikL.FlavellR. A.HanssonG. K. (2003). Disruption of TGF-beta signaling in T cells accelerates atherosclerosis. *J. Clin. Invest.* 112 1342–1350. 10.1172/JCI18607 14568988PMC228445

[B33] TakxR. A.PartoviS.GhoshhajraB. B. (2016). Imaging of atherosclerosis. *Int. J. Cardiovasc. Imaging* 32 5–12. 10.1007/s10554-015-0730-y 26239134

[B34] TianJ.LiuY.LiuY.ChenK.LyuS. (2017). Cellular and molecular mechanisms of diabetic atherosclerosis: herbal medicines as a potential therapeutic approach. *Oxid. Med. Cell Longev.* 2017:9080869. 10.1155/2017/9080869 28883907PMC5572632

[B35] WangY. Z.YangL.LiC. F. (2018). Protective effect of atorvastatin meditated by HMGCR gene on diabetic rats with atherosclerosis: an in vivo and in vitro study. *Biomed. Pharmacother.* 104 240–251. 10.1016/j.biopha.2018.04.179 29775891

[B36] WarnerD. R.HornK. H.MuddL.WebbC. L.GreeneR. M.PisanoM. M. (2007). PRDM16/MEL1: a novel Smad binding protein expressed in murine embryonic orofacial tissue. *Biochim. Biophys. Acta* 1773 814–820. 10.1016/j.bbamcr.2007.03.016 17467076

[B37] YeZ. M.YangS.XiaY. P.HuR. T.ChenS.LiB. W. (2019). LncRNA MIAT sponges miR-149-5p to inhibit efferocytosis in advanced atherosclerosis through CD47 upregulation. *Cell Death Dis.* 10:138. 10.1038/s41419-019-1409-4 30755588PMC6372637

[B38] YinH.PasutA.SoleimaniV. D.BentzingerC. F.AntounG.ThornS. (2013). MicroRNA-133 controls brown adipose determination in skeletal muscle satellite cells by targeting Prdm16. *Cell Metab.* 17 210–224. 10.1016/j.cmet.2013.01.004 23395168PMC3641657

[B39] ZhangR.SuiL.HongX.YangM.LiW. (2017). MiR-448 promotes vascular smooth muscle cell proliferation and migration in through directly targeting MEF2C. *Environ. Sci. Pollut. Res. Int.* 24 22294–22300. 10.1007/s11356-017-9771-1 28799067

[B40] ZhaoL.QiY.XuL.TaoX.HanX.YinL. (2018). MicroRNA-140-5p aggravates doxorubicin-induced cardiotoxicity by promoting myocardial oxidative stress via targeting Nrf2 and Sirt2. *Redox. Biol.* 15 284–296. 10.1016/j.redox.2017.12.013 29304479PMC5975069

[B41] ZhaoQ.SunD.LiY.QinJ.YanJ. (2019). Integrated analyses of lncRNAs microarray profiles and mRNA-lncRNA coexpression in smooth muscle cells under hypoxic and normoxic conditions. *Biosci. Rep.* 39:BSR20181783. 10.1042/BSR20181783 30850398PMC6443952

[B42] ZhuJ.LiuB.WangZ.WangD.NiH.ZhangL. (2019). Exosomes from nicotine-stimulated macrophages accelerate atherosclerosis through miR-21-3p/PTEN-mediated VSMC migration and proliferation. *Theranostics* 9 6901–6919. 10.7150/thno.37357 31660076PMC6815950

[B43] ZhuZ.WangH.WeiY.MengF.LiuZ.ZhangZ. (2017). Downregulation of PRDM1 promotes cellular invasion and lung cancer metastasis. *Tumour Biol.* 39:1010428317695929. 10.1177/1010428317695929 28378641

